# Empirical Analysis of Organization Quality-Specific Immune Evolution of Intelligent Manufacturing Enterprises Based on Self-Organization Methods

**DOI:** 10.1155/2022/6354820

**Published:** 2022-05-27

**Authors:** Qiang Liu, Yuqiong Tong, Danyu Zhao

**Affiliations:** School of Economics and Management, Liaoning University of Technology, Jinzhou 121001, China

## Abstract

Strengthening organization quality-specific immune is the key linkage to improve the quality performance of intelligent manufacturing enterprises. organization quality-specific immune is constructed by selecting four state variables of organization quality cognition, monitor, defense, and memory. Based on the perspective of self-organization, self-organization theory and methods are used to construct the evolution model of organization quality-specific immune. According to four state variables, the evolution of organization quality-specific immune of fourteen typical intelligent manufacturing enterprises is studied, and the conclusion is drawn according to the relaxation coefficient. The empirical results show that self-organization theory and self-organization methods can effectively analyze the evolution of organization quality-specific immune and provide new inspiration for organization quality improvement and quality management of intelligent manufacturing enterprises. The finding results will present the framework for practicing engineering managers of intelligent manufacturing enterprises to enhance organization quality performance and organization quality-specific immune performance and promote organization quality-specific immune evolution.

## 1. Introduction

Industry 4.0 advocates the fourth industrial revolution, transforms the manufacturing industry to intelligence, actively develops intelligent manufacturing enterprises, continuously improves the intelligence level of manufacturing enterprises, and promotes intelligent production, intelligent technology, human-computer interaction, intelligent management, intelligent network, and the intelligent resources of intelligent manufacturing enterprises. Quality is the core element of the intelligent manufacturing enterprise [1, 2]. Quality is the life of the intelligent manufacturing enterprise, the core element of organization management, and engineering management of intelligent manufacturing enterprise [3–8], and which is also the important strategic basis for enhancing sustainable competitiveness and development potential of intelligent manufacturing enterprise [9–20]. With the more prosperous life of people, people pay more attention to the pursuit of high-quality products; thus, improving the quality performance of intelligent manufacturing enterprises has become the most critical issue. However, various quality and safety problems still occur from time to time, and the incidents have aroused the attention of academic and practical fields and scopes. The vicious incidents not only damage the legitimate rights and interests of consumers but also have negative impacts on the long-term stability of intelligent manufacturing enterprises [21–26]. From the standpoints of medical immunology, a great many serious diseases are due to the fact that the body is exposed to the complex environment filled with bacteria, and the harmful bacteria and viruses are not effectively recognized, which will lead to immune behavior failure of the body and then cause the injury and death of the body. Therefore, the premise of healthy growth of the body is to improve and activate immune system function to improve the ability of the body to actively deal with and eliminate adverse factors. Nowadays, intelligent manufacturing enterprises exist in the complex environment full of bacteria-like organisms, and enterprises inevitably suffer from the threat of internal and external malignant quality events, which will result in the decline in the quality performance of intelligent manufacturing enterprises [2]. In order to cope with the fierce market competition environment, enterprises need to constantly update the quality management process, strengthen multifield quality management cooperation, and shorten the product cycle, which also increases the risk of exposure to more bacteria. Therefore, it is urgent to improve organization quality-specific immune function and strengthen the organization quality-specific immune behavior of intelligent manufacturing enterprises; especially, the adaptive, acquired, and noncongenital organization quality-specific immune behavior based on their own conditions is the key to the healthy development of intelligent manufacturing enterprises. With the change and evolution of quality connotation and quality function, new quality management paradigms and new quality management modes (organization quality immune and organization quality-specific immune) have been derived, which can adapt to the development of quality innovation strategy and quality power strategy; drive intelligent manufacturing enterprises to adopt better quality management practices, measures, and activities; and continuously improve quality performance [27–34]. If enterprises want to develop well, it is particularly important to establish a set of organization quality-specific immune system that is suitable for the development of enterprises in accordance with their own characteristics [35]. Nelson and Winter studied the enterprise evolution from a dynamic point of view and found that evolution could make the enterprise innovate continuously and adapt to market changes and improve its own state [36]. The organization quality-specific immune is a system, and the ultimate goals and destinations of organization quality-specific immune evolution lie in enhancing the quality performance of intelligent manufacturing enterprises. The evolution of organization quality-specific immune can make the structure and function of the organization immune system more complete. In addition, organization quality-specific immune of the intelligent manufacturing enterprise is under open and nonlinear conditions, and these conditions are in line with the evolution of self-organization. Self-organization theory and methods are a kind of evolution, and using the perspective of self-organization to study the evolution of enterprise system can provide us with a broader field of vision. Based on the perspective of self-organization theory and methods, this study constructs the evolution model of organization quality-specific immune; organization quality-specific immune is a system; organization quality-specific immune is composed of four construction elements of organization quality cognition, organization quality monitor, organization quality defense, and organization quality memory and makes an empirical study on the evolution of organization quality-specific immune.

Scholars home and abroad adopt interdisciplinary research ideas and methods to transplant, integrate, and map immunology to the quality management field; derive analogy and metaphor research results; and generate the connotation, function, classification system, and construction elements of organization immune; organization immune includes organization-specific immune and organization nonspecific immune; organization-specific immune is the core architecture of organization immune [37–55]. Lv and Wang studied the mechanism of organization immune behavior, which can be used as a reference for the development of organization quality immune system and organization quality-specific immune system [45, 56]. Jiang and Xiong, Xiong and Feng, and Jiang mainly studied the model of organization immune response [57–59]. Shi et al. studied the relationships between organization quality-specific immune and quality performance from the perspective of components consistency of organization quality-specific immune system [52]. Yang and Li paid attention to the problems encountered in the development of the organization by setting organization healthy development as the starting points [60]. Dai and Ding established the immune evaluation system based on the characteristics of self-enterprise immunity [61]. Through the analysis, it is found that scholars at home and abroad mainly analyze organization quality-specific immune through system structure, system function, and function mechanism based on the interdisciplinary research ideas and methods of organization immune. There is a lack of quantitative methods to carry out empirical analysis on the evolution of organization quality-specific immune. Therefore, this study constructs the evolution model of organization quality-specific immune; organization quality-specific immune is composed of four construct elements of organization quality cognition, organization quality monitor, organization quality defense, and organization quality memory by drawing lessons from absorbing a large number of relevant literature. This study further carries out an empirical analysis of the evolution and dynamic change tendency of organization quality-specific immune of intelligent manufacturing enterprises based on the perspective of self-organization; empirical analysis results will provide reference for practicing engineering managers and intelligent manufacturing enterprises to improve organization quality-specific immune performance and guide organization quality-specific immune evolution of intelligent manufacturing enterprises.

## 2. Literature Review

Quality is the life of intelligent manufacturing enterprise, on the basis of relevant research results of organization immune [37–55, 62]; organization quality immune is generated, organization quality immune includes organization quality-specific immune and organization quality nonspecific immune, and organization quality-specific immune is the core framework of organization quality immune [1]. Scholars at home and abroad have researched on the relevant contents and framework of organization quality-specific immune by theoretical and empirical research methods [41–52].

By drawing lessons from the relevant theoretical concepts of biological immunology, the scholars put forward the definition of organization quality immune, that is, enterprises find out the harmful factors that threaten product quality and organizational health, take the initiative and take immunization measures to deal with and eliminate the factors that threaten the quality, and generate the memory function as for the immunization process at the same time, in order to maintain the whole process healthy, quality performance, and stable development of enterprise [2, 21–26, 35, 36, 45, 52, 57–63]. Organization quality immune consists of organization quality-specific immune and organization quality nonspecific immune. Organization quality nonspecific immune is vital to the healthy development of enterprise quality, through which enterprises can filter most of the factors that endanger the quality safety and health of enterprises, which is the general and foremost immune behavior of enterprises to deal with the threatening factors including organization quality culture, organization structure, organization quality institution and rule, and organization quality resource [2, 21–26, 35, 36, 45, 52, 57–63]. Organization quality-specific immune is an important magic weapon for enterprises to maintain the quality stability, quality safety, and quality health. When enterprises are violated by threat factors, they can find negative factor in time and deal with and eliminate threat factor in time combined with their own quality characteristics [2, 21–26, 35, 36, 45, 52, 57–63]. Organization quality cognition, organization quality monitor, organization quality defense, and organization quality memory constitute organization quality-specific immune, and organization quality-specific immune is the core component of organization quality immune system [2, 21–26, 35, 36, 45, 52, 57–63]. Organization quality cognition is the process in which enterprises discover and identify harmful factors. There are differences in the cognition of threatening factors among different organizations. The occurrence of organization cognition behavior is a signal of immune behavior [42–44, 48–52, 63, 64]. Organization quality cognition is very important to the stable and healthy development of product quality of intelligent manufacturing enterprises on the cognition level [44, 51]. Organization quality monitor is to supervise the organization quality environment on the basis of organization quality cognition. Through organization quality monitor, we can find out the development trend and problems in the organization development stages in time [42, 43]. Organization quality defense is the process of organization to resist, eliminate, and renovate harmful factors of organization quality. Organization quality defense includes three steps of variation, selection, and coordination, which is the key of organization quality-specific immune [42–44, 48–52, 63, 64]. Organization quality memory refers to the whole process of improving organization quality-specific immune performance of enterprises through a series of immune behaviors of quality cognition, quality monitor, and quality defense, resulting in the accumulation of organization quality immunization knowledge base, including quality information, record, preservation, summary, diffusion, experience, and schemes [42–44, 48–52, 63, 64].

Through the analysis, it is found that scholars at home and abroad mainly analyze organization quality-specific immune through system structure, system function, and function mechanism according to organization immune. There is a lack of qualitative and quantitative methods to probe into the evolution of organization quality-specific immune. Therefore, this study constructs theoretical framework of organization quality-specific immune evolution model; organization quality-specific immune is composed of four construct elements of organization quality cognition, organization quality monitor, organization quality defense, and organization quality memory by drawing lessons from absorbing a large number of relevant literature and conducts empirical analysis of organization quality-specific immune evolution model according to self-organization methods.

## 3. Conceptual Framework of Organization Quality-Specific Immune Evolution

Organization quality-specific immune refers to the systematic concept, which is a system. Organization quality-specific immune is divided into four components of organization quality cognition, organization quality monitor, organization quality defense, organization quality memory, which can dominate and determine the evolution of organization quality-specific immune [27–31, 41–52, 56].

Organization quality cognition includes two parts of perception and discovery. The organization subject collects the object and quality-related information actively through organization quality cognition behavior, which is the expression form of organization initiative consciousness [52]. Through the screening and analysis of the internal and external information of organization, organization quality cognition can find out the factors that are disadvantageous to organization quality in time, deal with and delete the unfavorable factors in advance, and generate organization quality defense programs that adapt to the characteristics of the situation in order to maintain the stable development of enterprise [50]. Through the awareness of organization quality, enterprise managers can timely identify quality problems and effectively avoid risks and make reasonable strategic arrangements to improve quality performance [65, 66]. Lv and Wang suggested that the organization was a complex system, which was in the complex environment full of bacteria, and organization quality cognition was very important for enterprises to avoid risks and improve quality performance because different organizations had different degrees of complex environment cognition [42–44, 67]. Awareness of organization quality should be constantly updated and adapted to environmental development [68]. The perception of organization quality is the key for intelligent manufacturing enterprise to make the correct strategic plan. Kiesler and Sproull indicated that the key to organization immune behavior is to respond to the factors that stimulate organization, and the recognition of stimulus and motivation to deal with the factor is the premise of the occurrence of organization quality-specific immune [69]. Therefore, improving organization quality cognition plays a positive role in the evolution of organization quality-specific immune.

Organization quality monitor is an important link, and it is an important tool for senior managers to detect damage to product quality and health in time. The tool can help the enterprise to monitor the quality environment all the time so that the enterprise has been in a stable quality environment [52]. Through quality monitoring process, the enterprise can find the bad factors that affect product quality in time and restrain the occurrence of bad factors in time [56]. Organization quality monitor is a means for enterprises to control quality information. The senior managers of enterprises can grasp the changes of quality environment at any time, update quality information in time, and improve products' quality of enterprise. According to the results of monitoring, enterprise managers make favorable measures to product quality of enterprises and make corresponding decisions to make enterprises better adapt to the changing quality environment and improve products' quality. Organization quality monitor is an effective guarantee of product quality of intelligent manufacturing enterprise. By monitoring the organization environment at all times, enterprise managers can find out the quality problems existing in the organization in time, find the factors that threaten the quality, eliminate the enterprise quality problems in the initial stage, and further avoid risks in time. The enterprise makes the adjustment reasonably to formulate the optimal quality treatment plan and effectively reduces quality cost. With the increasing complexity of the market environment, the internal and external unfavorable factors of enterprises are also changing from time to time, so organization quality monitor should continue to evolve to adapt to the environment development. Therefore, organization quality monitor has a positive effect on the evolution of organization quality-specific immune.

Organization quality defense mainly includes three parts of variation, selection, and coordination. The defense process is carried out on the basis of effective monitoring of the organism, which refers to the process that the organization actively eliminates harmful factors of affecting quality in the organism [56]. Defense process is a continuous process, enterprises find adverse factors of product quality of intelligent manufacturing enterprises through monitoring behavior firstly, and then, enterprises timely activate and renew the occurrence of immune behavior according to the results of surveillance and deal with the exclusion of adverse factors. At the same time, through the comprehensive reference to the results of variation and selection, the organization coordinates the quality management practice and quality defense plan, selects the accurate countermeasures and suggestions, quickly forms the immune network, and improves product quality performance of intelligent manufacturing enterprises [70]. Organization quality defense is a process in which the enterprise subjectively removes the unfavorable factors of quality, and it is a reasonable defense behavior made by the enterprise according to the quality problem, which effectively reduces the emergence of enterprise quality crisis. Ferrier, Smith, and Grimm indicated that enterprises must take active and effective behavior to make enterprises adapt to the market environment and internal quality environment, and the organization quality defense behavior should also adapt to the market environment and internal quality environment, constantly carry out the quality defense evolution in order to timely, and accurately and quickly remove the factors that threaten product quality of intelligent manufacturing enterprise. Through the defense process, combined with the results of organization quality monitor, the results of defense are fed back to the organization, resulting in a series of immune behavior. Organization quality defense is the integration of a series of immune behavior [71]. March and Simon suggested that organization quality defense was very important to organization immune, and the enterprise separated, repaired, and cleared up adverse factors to form a whole set of organization quality defense system [72]. Therefore, organization quality defense is vital to the evolution performance of organization quality-specific immune.

Organization quality memory is the whole process of summarizing and digesting the immune process through memory behavior after a series of immune behavior [41]. The memory process is an effective means for enterprises to store quality-related knowledge. The defense scheme generated by enterprise will be effectively integrated into internal quality culture to help enterprise store quality information and knowledge, share quality experience, and establish their own quality database. Through memory behavior, enterprises can continue to learn quality knowledge in the process of immunization, summarize the experience of quality immunization, and record the quality-related knowledge at any time, and diffuse quality immunization knowledge. It is a tool for enterprise managers to store immune processes so that the relevant defense information can be integrated and summarized and become strategic objectives, working practices, and production rules of enterprises. At the same time, organization quality memory helps enterprises to make correct choices in the complex quality environment and maintain the stability of organization quality-specific immune performance. The organization can effectively record and summarize quality knowledge and improve the process of organization quality memory through organization quality memory tools. When the organism receives the antigen invasion, the immune behavior is produced by the organism, and the immune process can be recorded through the process. Therefore, organization quality memory can promote the evolution of organization quality-specific immune.

## 4. Methodology

### 4.1. Self-Organization Methods

Self-organization mainly studies the self-motion process of how the related subsystems of the system integrate into the regular structure [41, 73]. The occurrence of self-organization needs to meet the following conditions: (1) openness: that is, the system that can produce spontaneous and orderly behavior, and the system must be open. (2) Nonequilibrium: nonequilibrium is very important to self-organization behavior. The basic condition of order is nonequilibrium. (3) Nonlinear: nonlinearity is very important to self-organization, and the subsystem spontaneously becomes an ordered system through nonlinear action. Physicist Ha first put forward the concept of self-organization [74]. Ha found that the main source of power for the evolution of the system was the synergy and competition among the subsystems, and when the subsystems deviated from the original law, they behaved in an orderly manner [74]. When the system deviates from the original law of motion, the fluctuation phenomenon will be formed. This status quo is infinitely magnified to form a great driving force to promote the system to an orderly state. A great many scholars applied self-organization methods to the development of philosophy, management, economy, and other fields [75]. Self-organization is without any interference, and the system can obtain the complete structure. Self-organization itself is a kind of evolution, and using the perspective of self-organization to study the evolution and dynamic change tendency of enterprise system will provide a broader field of vision for researchers to probe into the evolution process among systems and subsystems from the perspective synergy theory [76]. Self-organization methods can be used in identifying the key influencing factors, order parameters, and slow variables that dominate the benign development and positive evolution of system, which can comprehensively probe into the evolution process, evolution path trend, and development tendency of the system [77–85].

### 4.2. Construction Principles and Steps of Evolution Model

#### 4.2.1. Construction Principles of Evolution Model

The principle of self-organization refers to the evolution theory within the system, which itself is a form of evolution [74]. Self-organization refers to hybrid methods. Based on the self-organization principle, through determining the research scope, the order parameters are found and the internal evolution mechanism of the system is found to analyze the influencing factors of the system evolution. Evolution is a periodic process, which is the result of the mutual promotion of related factors, and the competition among factors is the main driving force of evolution. The core theory of self-organization holds that the direct driving force of system development is the competition and synergy within the enterprise. Synergetics sets synergy and competition as the driving force of system evolution. Due to the existence of coordination and competition, some subsystems have great impacts on the organization, while others have smaller impacts [75].

The organization quality-specific immune is a system, it is necessary to explore the organization quality-specific immune from the perspective of the system. In this study, the relevant theory and methods of self-organization are used to study the evolution process. The scope of the research system and degree of grey correlations between the calculations are determined to find out the order parameters of the system [65, 74, 75]. According to the basic principle of self-organization evolution, the main power source of system evolution is the synergy and competition among subsystems [86–96]. When the system deviates from the original law of motion, the fluctuation phenomenon will be formed. This status quo is infinitely magnified to form a great driving force to promote the system to an orderly state.

#### 4.2.2. Construction Steps of Evolution Model

The steps of constructing the evolution model are as follows [86–96]:

(1) *Determining the Order Parameters of the System*. The order parameter is a parameter at the macrolevel, and the order parameter can better express the behavior of the system. Order parameters are mainly used to express the disordered and ordered state of the system. Its core is the change of two phases after the phase transition occurs, and the order parameter is to describe the different physical quantities between two phases. The order parameters determine the direction of system evolution. Ha introduced the concept of order parameters into synergetics knowledge, that is, the variables that discovered and determined the formation and evolution of the system [74]. Ha believed that the order parameters played vital roles in the evolution of the system, which dominated the overall trend of the system evolution [74]. In summary, the order parameters determine the direction of system evolution, the evolution of the system is the result of the coordination and competition of each subsystem and elements of the subject, and different elements have different effects on the whole evolution system.
(2) *Determining the State Variables*. State variables are designed to better outline the variables of the system in a state. According to the state variables, the evolution equation of the research system is established based on the model method, and the order parameters are determined at the same time. According to the research purpose of the system and each subsystem, the state variables are selected reasonably.
(3) *Calculating the Correlation Degree of Subsystem Variables*. First of all, the grey correlation degree is calculated, and the correlation degree of each variable is obtained according to the numerical value; thus, the state variable of the system is obtained. The basic idea of grey relational analysis is to use the quantitative method to determine the quantity of variables in the system and then judge the degree of correlation among the variables [66]. According to the sequence image of system to analyze the correlation of related factors, the degree of image similarity is large, indicating that the factors are closely related; the smaller the image similarity is, the smaller the correlation among the factors is.
(4) *Dimensionless Processing of Data*. Each variable cannot hold on to its unique economic meaning, and the dimensionless nature of the data is to eliminate the difference [65]. It can be done as long as there are dimensional variables. Through the process, the calculation steps are effectively simplified. Through the dimensionless processing of the system data, it can better enhance the comparability between the data.
(5) *Processing the Data by Accumulation and Generation*. The main process of generating and processing the accumulation of data is the process of accumulating different data to obtain a new sequence of numbers. This method can make the data of the system change from grey to white so that the unique law of invisibility between data without any law can be manifested [66].
  (1) $$\begin{array}{c} X_{i}^{\left(1\right)}\left(k\right)=\overset{t=k}{\underset{t=1}{\sum }}X_{i}^{\left(0\right)}\left(t\right). \end{array}$$
(6) *Establishing Differential Equation and Measurement Analysis Results*. There is external synergy among the research factors of organization quality-specific immune in the system, which is the result of coordination and competition, and the cooperative items are *aijx*_*j*_^(1)^(*t*), *a*_*ij*_≻0 represents the synergistic effect of *j* element on *i* element; *a*_*ij*_≺0 represents the competitive effect of *j* element on *i* element. As a result, the total rate of change of *X*_*i*_^(1)^(*t*) is as follows:

(2) $$\begin{array}{c} \frac{\text{d}X_{i}^{\left(1\right)}\left(t\right)}{\text{d}t}=aiix_{i}^{\left(1\right)}\left(t\right)-bii{\left(X_{i}^{\left(1\right)}\left(t\right)\right)}^{2}+\overset{n}{\underset{j=1j\neq 1}{\sum }}a_{ij}x_{i}^{\left(1\right)}\left(t\right)+f_{i}\left(t\right), \end{array}$$

where the synergy is expressed as *bijx*_*j*_^(1)^(*t*), the competitive effect is expressed as *aij*(*X*_*j*_^(1)^(*t*))^2^, *f*_*i*_(*t*) refers to external interference factors. −*b*_*ii*_=*b*_*i*_, then the nonlinear equation can be reduced to

(3) $$\begin{array}{c} \frac{\text{d}X_{i}^{\left(1\right)}\left(t\right)}{\text{d}t}=aiX_{i}^{\left(1\right)}\left(t\right)+bi{\left(X_{i}^{\left(1\right)}\left(t\right)\right)}^{2}+\overset{n}{\underset{j=1j\neq 1}{\sum }}\left(a_{ij}x_{j}^{\left(1\right)}\left(t\right)+f_{i}\left(t\right)\right). \end{array}$$

According to the principle of least square method, *y*=min∑_*t*=2_[*x*_*i*_^(0)^(*t*) − *b*_*i*_[*x*_*i*_^(1)^(*t*)]^2^ − 4∑_*j*=1_^4^*a*_*ij*_*x*_*j*_^(1)^(*t*)]^2^. According to the extreme value condition of multivariate function, the conclusion is drawn.

## 5. Empirical Analysis

### 5.1. Order Parameters of Organization Quality-Specific Immune Evolution

There are various multiple relationships among the internal factors of organization quality-specific immune. To study its evolution system, it is necessary to analyze the scope of organization quality-specific immune and get the correlations among the factors so as to find out the order parameters of the system accurately.

### 5.2. State Variables of Organization Quality-Specific Immune Evolution

State variables of organization quality-specific immune evolution refer to organization quality cognition, organization quality monitor, organization quality defense, and organization quality memory.

### 5.3. Determining the Correlation Degree of Subsystem Variables

According to the evolution model, we calculate the grey correlation degree and get the correlation degree of each variable according to the numerical value so as to get the state variable of the system. In this study, fourteen representative large-scale intelligent manufacturing enterprises in eastern China are taken as the evaluation objects, and four subsystems are constructed, including organization quality cognition, monitor, defense, and memory. This study makes out dynamic evaluation on the organization quality-specific immune evolution of intelligent manufacturing enterprises in eastern China.

By the form of on-site distribution questionnaire, fourteen representative benchmark intelligent manufacturing enterprises (*X*_1_–*X*_14_) in eastern China are selected as samples. The questionnaire is divided into two parts of the basic information of the object and the score of the questionnaire. Among them, the basic information part of the survey object requires the survey object to fill in the personal information, and the scoring part will affect the four state variables and further affect the evolution of the system. This study uses organization quality cognition *C*_1_, organization quality monitor *C*_2_, organization quality defense *C*_3_, and organization quality memory *C*_4_ to score. Among them, 1–2 indicates weak influence on the evolution of organization quality-specific immune, 3–5 indicates average influence, 5–6 indicates higher influence, and 7–8 indicates strong influence.

The first step is the preinvestigation and developing formal questionnaire stage. The maneuverability of the questionnaire is pretested before issuing the questionnaire, and the middle and senior managers of typical benchmarking intelligent manufacturing enterprises, staff, personnel, and relevant experts are invited to analyze and modify the accuracy, maneuverability, and representativeness of the questionnaire. The second step is the formal investigation stage, and we develop formal questionnaires by on-site distribution questionnaire. A total of 480 questionnaire vouchers are issued in this survey, of which 415 questionnaires are collected and 58 questionnaires are invalid, with an effective rate of 74.37%. Processing and analyzing the effective questionnaire, using SPSS25.0 software to test the reliability of the effective questionnaire, Cronbach's Alpha value is 0.795, indicating that the internal consistency of the various variables is high and the reliability is good. After that, the validity of the collected effective questionnaire is calculated, and it is concluded that the KMO value is 0.765 > 0.7, and the validity is less than 0.001. It shows that the content of this survey captures the main characteristics of the questionnaire. The questionnaire, scale, and the collected data can effectively achieve the purpose of the investigation. Among the 357 valid questionnaires, the following conclusions are drawn: most of the respondents are men, accounting for 64%, and the age distribution is between 35 and 50 years old, accounting for 85%. As for education, 57% is undergraduate course. As for working years, 62% is 10–15 years, 17% is less than 10 years, and 21% is more than 15 years. According to the scoring situation, the data of valid questionnaire are average processed by SPSS25.0 software, and the average results are used as the original values of related variables as shown in Table 1.

Through the grey relational analysis and calculation [65], the grey correlation degree of each state variable is shown in Table 2.

As for the 357 valid questionnaires, it can be concluded from the grey correlation values of state variables in Table 2 that the four state variables can affect the evolution of organization quality-specific immune of intelligent manufacturing enterprises, the four state variables support and restrict each other, and the correlation degree is obvious. The related test results indicate that the interactions among four state variables are nonlinear, coupled, and cooperative.

### 5.4. Dimensionless Processing of Data

According to the empirical analysis of the evolution model, the fourth step is dimensionless treatment. The specific calculation formula is as follows [65, 66]:

(4) $$\begin{array}{c} X_{i}^{\left(0\right)}\left(t\right)=\frac{X_{i}\left(t\right)-\underset{t}{\min}X_{i}\left(t\right)}{\underset{t}{\max}X_{i}\left(t\right)-\underset{t}{\min}X_{i}\left(t\right)}. \end{array}$$

Let variable *X*_*i*_(*t*) represent the data (*i*=1,2,3,4;  *t*=1,2,…, 14) of the first index of the *t* enterprise, and the data sequence after dimensionless processing is *X*_i_^(0)^(*t*)(*i*=1,2,3,4, *t*=1,2,…, 14) as shown in Table 3.

### 5.5. Data Processing by Accumulation and Generation

According to construction steps of the evolution model, we carry out the accumulation and generation processing to the data, and specific data are shown in Table 4. The specific formula is as follows:

(5) $$\begin{array}{c} X_{i}^{\left(1\right)}\left(k\right)=\overset{t=k}{\underset{t=1}{\sum }}X_{i}^{\left(0\right)}\left(t\right). \end{array}$$

*X*_*i*_^(*t*)^(*i*=1,2,3,4, *t*=1,2,…, 14) is treated with AGO and recorded as *X*_*i*_^(1)^(*t*) [75, 76, 97].

### 5.6. Differential Equation Establishment

The change of *X*_*i*_^(1)^(*t*) derives from two factors, one is the internal synergy, and the other is the external synergy among the various elements. Internal synergy refers to the result of its own development and self-inhibition [65, 66]. Through the grey correlation analysis, it can be concluded that the internal synergy is nonlinear. In order to make the analysis process simple and reasonable, it is assumed that the internal synergy is a quadratic curve, so the self-development term is *aix*_*i*_^(1)^(*t*) and the self-inhibition term is *aix*_*i*_^(1)^(*t*). The rate of change is affected and disturbed by other factors of its own development [97]. In the model, *aix*_*i*_^(1)^(*t*) is the self-development ability of the *i* state variable, and *a*_*i*_ represents for the coefficient of the state parameter, that is, the relaxation coefficient [68].

The external synergy among the system elements is recorded as *aijx*_*j*_^(1)^(*t*); *a*_*ij*_≻0 represents the synergy of *j* elements to *i* elements; *a*_*ij*_≺0 represents the competitive effect of *j* elements on *i* elements. As a result, the total rate of change of *X*_*i*_^(1)^(*t*) is [65, 95, 96]

(6) $$\begin{array}{c} \frac{\text{d}X_{i}^{\left(1\right)}\left(t\right)}{\text{d}t}=aiix_{i}^{\left(1\right)}\left(t\right)-bii{\left(X_{i}^{\left(1\right)}\left(t\right)\right)}^{2}+\overset{n}{\underset{j=1j\neq 1}{\sum }}a_{ij}x_{i}^{\left(1\right)}\left(t\right)+f_{i}\left(t\right), \end{array}$$

∑_*j*=1*j*≠1_^*n*^[(*b*_*ij*_*x*_*j*_^(1)^(*t*)+*a*_*ij*_(*X*_*j*_^(1)^(*t*))^2^] represents the synergistic and competitive effect of state variables on *i* variables.

Among them, the synergy is expressed as *b*_*ij*_*x*_*j*_^(1)^(*t*); the competition is expressed as *a*_*ij*_(*X*_*j*_^(1)^(*t*))^2^; *f*_*i*_(*t*) represents the external interference factors. −*b*_*ii*_=*b*_*i*_, then the nonlinear equation can be deduced to

(7) $$\begin{array}{c} \frac{\text{d}X_{i}^{\left(1\right)}\left(t\right)}{\text{d}t}=a_{i}X_{i}^{\left(1\right)}\left(t\right)+b_{i}{\left(X_{i}^{\left(1\right)}\left(t\right)\right)}^{2}+\overset{n}{\underset{j=1j\neq 1}{\sum }}\left(a_{ij}x_{j}^{\left(1\right)}\left(t\right)+f_{i}\left(t\right)\right). \end{array}$$

Assuming that d*X*_*i*_^(1)^(*t*)/d*t*=*X*_*i*_^(1)^(*t*) − *X*_*i*_^(1)^(*t* − 1)=*X*_*i*_^(0)^(*t*).

(8) $$\begin{array}{c} \frac{\text{d}X_{i}^{\left(1\right)}\left(t\right)}{\text{d}t}=bi{\left(X_{i}^{\left(1\right)}\left(t\right)\right)}^{2}+\overset{4}{\underset{j=1j\neq 1}{\sum }}\left(\left(aijX_{j}^{\left(1\right)}\left(t\right)\right)+f_{i}^{\left(t\right)}\right),\\ f_{i}\left(t\right)=x_{i}^{\left(0\right)}\left(t\right)-b_{i}{\left[x_{i}^{\left(1\right)}\left(t\right)\right]}^{2}-{\overset{4}{\underset{j=1}{\sum }}a_{ij}x_{j}}^{\left(1\right)}\left(t\right). \end{array}$$

According to the principle of least square method, it can be concluded as follows:

(9) $$\begin{array}{c} y=\min{\overset{14}{\underset{t=2}{\sum }}\left[x_{i}^{\left(0\right)}\left(t\right)-b_{i}{\left[x_{i}^{\left(1\right)}\left(t\right)\right]}^{2}-\overset{4}{\underset{j=1}{\sum }}a_{ij}x_{j}^{\left(1\right)}\left(t\right)\right]}^{2}. \end{array}$$

According to the extreme value condition of multivariate function, it can be concluded as follows:

(10) $$\begin{array}{c} \frac{\partial y}{\partial b_{i}}=-2\overset{14}{\underset{t=2}{\sum }}\left[x_{i}^{\left(0\right)}\left(t\right)-b_{i}{\left[x_{i}^{\left(1\right)}\left(t\right)\right]}^{2}-\overset{4}{\underset{j=1}{\sum }}a_{ij}x_{j}^{\left(1\right)}\left(t\right)\right]{\left[x_{i}^{\left(1\right)}\left(t\right)\right]}^{2},\\ =-2\overset{14}{\underset{t=2}{\sum }}\left[x_{i}^{\left(0\right)}\left(t\right){\left[x_{i}^{\left(1\right)}\left(t\right)\right]}^{2}-b_{i}{\left[x_{i}^{\left(1\right)}\left(t\right)\right]}^{4}-\overset{4}{\underset{j=1}{\sum }}a_{ij}x_{j}^{\left(1\right)}\left(t\right){\left[x_{i}^{\left(1\right)}\left(t\right)\right]}^{2}\right],\\ \frac{\partial y}{\partial a_{ik}}=-2\overset{14}{\underset{t=2}{\sum }}\left[x_{i}^{\left(0\right)}\left(t\right)-b_{i}{\left[x_{i}^{\left(1\right)}\left(t\right)\right]}^{2}-\overset{4}{\underset{j=1}{\sum }}a_{ij}x_{j}^{\left(1\right)}\left(t\right)\right]{\left[x_{k}^{\left(1\right)}\left(t\right)\right]}^{2},\\ =-2\overset{14}{\underset{t=2}{\sum }}\left[x_{i}^{\left(0\right)}\left(t\right)x_{k}^{\left(1\right)}\left(t\right)-b_{i}{\left[x_{i}^{\left(1\right)}\left(t\right)\right]}^{2}x_{k}^{\left(1\right)}\left(t\right)-\overset{4}{\underset{j=1}{\sum }}a_{ij}x_{j}^{\left(1\right)}\left(t\right)x_{k}^{\left(1\right)}\left(t\right)\right]. \end{array}$$

Substitute *t*=2,3,…, 14, separate into the above formula, *y*_*N*_=*B*_*i*_*P*_*i*_.

(11) Bi=∑t=214xi1t4∑t=214x11txi1t2∑t=214x21txi1t2∑t=214x31txi1t2∑t=214x41txi1t2∑t=214x11txi1t2∑t=214x11tx11t∑t=214x21tx11t∑t=214x31tx11t∑t=214x41tx11t∑t=214x21txi1t2∑t=214x11tx21t∑t=214xt21x21t∑t=214x31tx21t∑t=214x41tx21t∑t=214x31txi1t2∑t=214x11tx31t∑t=214x21tx31t∑t=214x31tx31t∑t=214x41tx31t∑t=214x41txi1t2∑t=214x11tx41t∑t=214x21tx41t∑t=214x31tx41t∑t=214x41tx41t,yi=∑t=2t=14xi0txi1t2∑t=2t=14xi0tx11t2∑t=2t=14xi0tx21t2∑t=2t=14xi0tx31t2∑t=2t=14xi0tx41t2,P=biai1ai2ai3ai4T.

### 5.7. Measurement Analysis

Replace the dimensionless data into *B*_*i*_ to obtain *B*_1_, *B*_2_, *B*_3_, and *B*_4_ and replace the cumulative added data into *y*_*i*_ to obtain *y*_1_, *y*_2_, *y*_3_, and *y*_4_; the results are as follows [86–96, 98]:

(12) $$\begin{array}{c} B_{1}=\left[\begin{array}{ccccc} 1948.707 & 451.1094 & 667.0625 & 501.0156 & 573.9375\\ 451.1094 & 112.8125 & 175.875 & 126.9375 & 152\\ 667.0625 & 175.875 & 286.3125 & 200.6875 & 246.8125\\ 501.0156 & 126.9375 & 200.6875 & 144.4375 & 173.1875\\ 573.9375 & 152 & 246.8125 & 173.1875 & 214.3125 \end{array}\right],\\ y_{1}=\left[\begin{array}{c} 52.4375\\ 14.25\\ 22.1875\\ 15.125\\ 19.4375 \end{array}\right]. \end{array}$$

Matrix B is a symmetric positive definite matrix, so there is a unique solution. The inverse matrix *B*^−1^ of *B* is obtained from the cumulative added data [98], and the concrete value is obtained by MATLAB software according to *P*_*i*_=*B*_*i*_^−1^ × *y*_*i*_.

(13) $$\begin{array}{c} P_{1}={\left[\begin{array}{ccccc} -0.1187 & 1.7480 & 0.0031 & -0.7462 & -0.2318 \end{array}\right]}^{T}. \end{array}$$

In the same way, we can obtain the following results:

(14) $$\begin{array}{c} B_{2}=\left[\begin{array}{ccccc} 9384.2227 & 1015.313 & 1600.5156 & 1150.922 & 1368.391\\ 1015.313 & 112.8125 & 185.875 & 126.9375 & 152\\ 1600.516 & 185.875 & 286.3125 & 200.6875 & 246.8125\\ 1150.922 & 126.9375 & 200.6875 & 144.4375 & 173.1875\\ 1368.391 & 152 & 246.8125 & 173.1875 & 214.3125 \end{array}\right]y_{2}=\left[\begin{array}{c} 148.2188\\ 15.9375\\ 28.5\\ 18.25\\ 24.3125 \end{array}\right],\\ P_{2}={\left[\begin{array}{ccccc} 0.0024 & 0.0982 & 0.5125 & -0.5670 & -0.1036 \end{array}\right]}^{T},\\ B_{3}=\left[\begin{array}{ccccc} 2967.168 & 560.5469 & 845.5469 & 632.0781 & 725.9219\\ 560.5469 & 112.8125 & 175.875 & 126.9375 & 152\\ 845.5469 & 175.875 & 286.3125 & 200.6875 & 246.8125\\ 632.0781 & 126.9375 & 200.6875 & 144.4375 & 173..1875\\ 725.921875 & 152 & 246.8125 & 173.1875 & 214.3125 \end{array}\right]y_{3}=\left[\begin{array}{c} 74.7656\\ 15.3125\\ 26\\ 18.4375\\ 22.4375 \end{array}\right],\\ P_{3}={\left[\begin{array}{ccccc} -0.0513 & -0.5747 & -0.1473 & 1.1552 & -0.0778 \end{array}\right]}^{T},\\ B_{4}=\left[\begin{array}{ccccc} 5071.0195 & 750.9688 & 1177.172 & 849.8281 & 1019.109\\ 750.9688 & 112.8125 & 175.875 & 126.9375 & 152\\ 117.1719 & 175.875 & 286.3125 & 200.6875 & 246.8125\\ 846.8281 & 126.9375 & 200.6875 & 144.4375 & 173.1875\\ 1019.109 & 152 & 246.8125 & 173.1875 & 214.3125 \end{array}\right]y_{4}=\left[\begin{array}{c} 74.5\\ 10.9375\\ 19.4375\\ 12.625\\ 18 \end{array}\right],\\ P_{4}={\left[\begin{array}{ccccc} -0.0167 & -0.1239 & -0.4987 & -0.0794 & 0.8899 \end{array}\right]}^{T}. \end{array}$$

### 5.8. Empirical Analysis Results

*C*_*i*_(*i*=1,2,3,4) is the relaxation coefficient of each index system in the organization quality-specific immune system. According to the coevolution model, the relaxation coefficient of each index system is obtained: *C*_1_ = 1.7480, *C*_2_ = 0.5125, *C*_3_ = 1.1552, and *C*_4_ = 0.8899. The relationships among the relaxation coefficients of each index system are as follows: *C*_2_ < *C*_4_ < *C*_3_ < *C*_1_.

The relaxation coefficient represents the influence degree of the state variable on the evolution of organization quality-specific immune, that is, the smaller the relaxation coefficient is, the greater the effect and influence on the evolution of organization quality-specific immune is, and the greater the relaxation coefficient is when the state variable has a slight effect on the evolution of organization quality-specific immune. According to the empirical analysis results, organization quality monitor has the greatest influence on the evolution of organization quality-specific immune, organization quality memory has the greater influence on the evolution of organization quality-specific immune, organization quality defense has a general influence on the evolution of organization quality-specific immune, and organization quality cognition has the least influence on the evolution of organization quality-specific immune.

## 6. Conclusions and Practical Implications

### 6.1. Conclusions

The related theory and methods of self-organization are introduced into the evolution model of organization quality-specific immune of intelligent manufacturing enterprises. With the help of self-organization theory and methods [65, 74], this study studies and analyzes the evolution process of organization quality-specific immune through the relevant theory of synergetics and explores the influencing factors of organization quality-specific immune evolution based on self-organization methods. This study constructs four subsystems of organization quality cognition, monitor, defense, and memory, then determines the order parameters of organization quality-specific immune evolution, makes out empirical analysis of the evolution of organization quality-specific immune, and finds out the influencing factors of organization quality-specific immune evolution. This study selects four state variables of organization quality cognition, organization quality monitor, organization quality defense, and organization quality memory and makes out on-site distribution questionnaire according to the influence of four state variables on organization quality-specific immune evolution. Fourteen representative benchmark intelligent manufacturing enterprises (large scale and major enterprises) in eastern China are selected as samples, the obtained data are treated as sample data for dimensionless processing and cumulative addition processing, and the relaxation coefficient is obtained after the empirical analysis of differential equation.

According to the relaxation coefficient, it is concluded that different state variables have different influences on the evolution of organization quality-specific immune, that is, organization quality monitor has the greatest effect on the evolution of organization quality-specific immune, organization quality memory has the greater influence on the evolution of organization quality-specific immune, organization quality defense has a general effect on the evolution of organization quality-specific immune, and organization quality cognition has the least effect on the evolution of organization quality-specific immune. It is urgent to enhance organization quality-specific immunity in accordance with local conditions on the weak points of the evolution of organization quality-specific immune [41]. The purpose of this study is to help enterprise managers to better manage organization quality-specific immune and take reasonable measures to improve the organization quality performance of intelligent manufacturing enterprise; provide new ideas for the theoretical and practical study of the evolution of organization quality-specific immune; improve the correlation relationships of the influencing factors of organization quality-specific immune evolution; better grasp different influence degrees; influence sequences and orders of organization quality monitor, organization quality memory, organization quality defense, and organization quality cognition in the process of organization quality-specific immune evolution; advocate and encourage organization quality monitor and organization quality memory positively; and strengthen and enhance organization quality defense and organization quality cognition significantly. This study has a certain theoretical guiding value and practical significance.

### 6.2. Practical Implications

The practical implications for engineering managers of intelligent manufacturing enterprises lie in the following:

1. Theoretical research framework of this study can be used by practicing engineering managers; engineering managers of intelligent manufacturing enterprises can understand the key role and significance of quality in the process of engineering management and organization management; comprehensively examine quality management problems from the perspective of immune; strengthen the soft and hard elements of quality management practice; activate the function and vitality of hard and soft elements of organization quality defense; develop institutional and social measures; focus on the core practice and basic practice of quality management; realize quality improvement cycle; form the virtuous cycle and context system of mutual promotion, coordination, correction, and feedback among organization quality cognition, organization quality monitor, organization quality defense, and organization quality memory; enhance organization quality trial and error ability; promote organization quality-specific immune evolution (genetic replication evolution, cross mutation evolution and adaptive development evolution); and improve organization quality competitiveness, quality innovation ability, quality management ability, customer satisfaction, organization operation efficiency, and organization finance performance
2. In terms of the theoretical research framework of this study, engineering managers of intelligent manufacturing enterprises can also judge and examine quality management issues from the perspective of system and evolution; put emphasis on the functions of organization quality cognition, organization quality monitor, organization quality defense, and organization quality memory; activate and dredge the function of organization quality-specific immune; prevent hypersensitivity and hyperimmunity; enhance organization quality-specific immune response rate; continuously increase quality performance and core competitiveness; improve organization quality improvement efficiency, market share, productivity, and final product quality qualification rate; and reduce product quality assurance cost, total quality cost, and quality defects compared with competitors
3. The empirical analysis results of this study can be applied by practicing engineering managers; engineering managers of intelligent manufacturing enterprises can recognize that organization quality-specific immune is a system; actively promote the orderly evolution of organization quality-specific immune; drive organization quality-specific immune to maintain the good evolution trend and development tendency; prompt the spiral upgrading, function optimization, and function renewal of organization quality-specific immune; introduce negative entropy flow; make organization quality-specific immune get into the virtuous cycle process and track; stimulate the niche change of organization quality system; enhance the maturity, survivability, robustness, disaster tolerance, and buffer capacity of organization quality-specific immune system; and reduce the vulnerability and redundancy of organization quality system
4. In terms of the empirical analysis results of this study, engineering managers of intelligent manufacturing enterprises can also identify the key factors, dominant slow variables, and order parameters of organization quality-specific immune evolution; emphasize on the obstacle factors and weak links of organization quality-specific immune development; excavate the bottleneck factors that hinder the evolution of organization quality-specific immune; refine the operation paths of organization quality-specific immune evolution according to the relevant parameters of organization quality cognition, organization quality monitor, organization quality defense, and organization quality memory; actively guide the evolution direction of organization quality system; and complete organization quality strategy and mission

## Figures and Tables

**Table 1:** Original values of state variables (average processed).

Status index	*X*_1_	*X*_2_	*X*_3_	*X*_4_	*X*_5_	*X*_6_	*X*_7_	*X*_8_	*X*_9_	*X*_10_	*X*_11_	*X*_12_	*X*_13_	*X*_14_
*C*_1_	4	3	6	3	4	3	6	4	5	4	7	3	7	3
*C*_2_	6	4	4	7	5	6	7	3	6	5	3	3	5	7
*C*_3_	3	6	3	5	3	5	5	7	3	4	6	5	4	6
*C*_4_	6	3	6	6	4	7	3	4	6	3	6	4	3	4

**Table 2:** Grey correlation table of state variables.

Status index	*C*_1_	*C*_2_	*C*_3_	*C*_4_
*C*_1_	1	0.725747	0.686484	0.703628
*C*_2_	0.725747	1	0.661489	0.795939
*C*_3_	0.686484	0.661489	1	0.654639
*C*_4_	0.703628	0.795939	0.654639	1

**Table 3:** Dimensionless data table.

Status index	*X*_1_	*X*_2_	*X*_3_	*X*_4_	*X*_5_	*X*_6_	*X*_7_	*X*_8_	*X*_9_	*X*_10_	*X*_11_	*X*_12_	*X*_13_	*X*_14_
*C*_1_	0.25	0	0.75	0	0.25	0	0.75	0.25	0.5	0.25	1	0	1	0
*C*_2_	0.75	0.25	0.25	1	0.5	0.75	1	0	0.75	0.5	0	0	0.5	1
*C*_3_	0	0.75	0	0.5	0	0.5	0.5	1	0	0.25	0.75	0.5	0.25	0.75
*C*_4_	0.75	0	0.75	0.75	0.25	1	0	0.25	0.75	0	0.75	0.25	0	0.25

**Table 4:** Data accumulation to generate numerical tables.

Status index	*X*_1_	*X*_2_	*X*_3_	*X*_4_	*X*_5_	*X*_6_	*X*_7_	*X*_8_	*X*_9_	*X*_10_	*X*_11_	*X*_12_	*X*_13_	*X*_14_
*C*_1_	0.25	0.25	1	1	1.25	1.25	2	2.25	2.75	3	4	4	5	5
*C*_2_	0.75	1	1.25	2.25	2.75	3.5	4.5	4.5	5.25	5.75	5.75	5.75	6.25	7.25
*C*_3_	0	0.75	0.75	1.25	1.25	1.75	2.25	3.25	3.25	3.5	4.25	4.75	5	5.75
*C*_4_	0.75	0.75	1.5	2.25	2.5	3.5	3.5	3.75	4.5	4.5	5.25	5.5	5.5	5.75

## Data Availability

The data sets used and/or analyzed during the current study are available from the corresponding author on reasonable request.

## References

[1] Liu Q., Qu X., Zhao D., Guo Y. (2021). Qualitative simulation of organization quality-specific immune decision-making of manufacturing enterprises based on QSIM algorithm simulation. *Journal of Computational Methods in Science and Engineering*.

[2] Xu H., Ji C. L., Li J. (2011). Research on risk response mechanism of science and technology small and medium-sized enterprises from the perspective of organization immune. *Management World*.

[3] Blessner P., Mazzuchi T. A., Sarkani S. (2013). ISO 9000 impact on product quality in a defense procurement environment. *The TQM Journal*.

[4] Chao G. H., Iravani S. M. R., Savaskan R. C. (2009). Quality improvement incentives and product recall cost sharing contracts. *Management Science*.

[5] Garstenauer A., Blackburn T., Olson B. (2014). A knowledge management based approach to quality management for large manufacturing organizations. *Engineering Management Journal*.

[6] Haq S. U., Liang C., Gu D., Du J. T., Zhao S. (2018). Project governance, project performance, and the mediating role of project quality and project management risk: an agency theory perspective. *Engineering Management Journal*.

[7] Linderman K., Schroeder R. G., Zaheer S., Liedtke C., Choo A. S. (2004). Integrating quality management practices with knowledge creation processes. *Journal of Operations Management*.

[8] Shan S., Zhao Q., Hua F. (2013). Impact of quality management practices on the knowledge creation process: the Chinese aviation firm perspective. *Computers & Industrial Engineering*.

[9] Agyabeng-Mensah Y., Ahenkorah E., Afum E., Qwusu D. (2020). The influence of lean management and environmental practices on relative competitive quality advantage and performance. *Journal of Intelligent manufacturing Technology Management*.

[10] Dellana S. A., Coffin M. A. (1996). Quality management tactics in U.S. Manufacturing: do they rival the Japanese?. *Engineering Management Journal*.

[11] Feng L., Huang D., Jin M., Li W., He Z., Yu A. J. (2020). Quality control scheme selection with a case of aviation equipment development. *Engineering Management Journal*.

[12] Harris E. D., Koshy T., Anderson R. L. (2015). Concurrent engineering and total quality management: the need for a seamless marriage. *Engineering Management Journal*.

[13] Milunovic Koprivica S., Filipovic J. (2018). Application of traditional and fuzzy quality function deployment in the product development process. *Engineering Management Journal*.

[14] Lee V. H., Foo P. Y., Tan G. W. H., Ooi K. B., Sohal A. (2021). Supply chain quality management for product innovation performance: insights from small and medium-sized intelligent manufacturing enterprises. *Industrial Management & Data Systems*.

[15] Marion J. W., Richardson T. M., Anantatmula V. (2021). Managing quality in aviation projects. *Engineering Management Journal*.

[16] Ruso J., Glogovac M., Filipović J., Jeremić V. (2021). Employee fluctuation in quality management profession: exploiting social professional network data. *Engineering Management Journal*.

[17] Tarí J. J., Molina-Azorín J. F., Pereira-Moliner J., López-Gamero M. D. (2020). Internalization of quality management standards: a literature review. *Engineering Management Journal*.

[18] Utley D. R., Westbrook J., Turner S. (1997). The relationship between Herzberg’s two-factor theory and quality improvement implementation. *Engineering Management Journal*.

[19] Wan X., Li D., Chen J., Lei Y. (2020). Managing customer returns strategy with the option of selling returned products. *International Journal of Production Economics*.

[20] Zhou H., Li L. (2020). The impact of supply chain practices and quality management on firm performance: e. *International Journal of Production Economics*.

[21] Cui Y. J., Li Y. X., Chen K. J. (2018). The impact of external governance environment on earnings quality: is natural resource endowment a curse?. *Nankai Business Review*.

[22] Han C., Zhu P. Z. (2018). The evolution of foreign investment access policy and its impact on the quality of intelligent manufacturing products since the reform and opening up. *Management World*.

[23] Hua F. T., Xu F. (2018). How does environmental uncertainty affect corporate idiosyncratic risk-An mediating effect test based on cash flow fluctuation and accounting information quality. *Nankai Business Review*.

[24] Li T., Dong Y. M., Wang Z. Y. (2018). Management efficiency, quality ability and total factor productivity of enterprises-An empirical study based on “Chinese enterprise-labor force matching survey”. *Management World*.

[25] Pan X. W., Wang N. (2015). Research on the principle and ability improvement path of enterprise quality immune response. *Journal of Chongqing Jianzhu University*.

[26] Ren H. D., Wang K. (2018). Social relations and the quality of enterprise information disclosure-A text analysis based on the annual report of Chinese listed companies. *Nankai Business Review*.

[27] Liu Q., Hu H., Guo Y. (2020). Organizational quality specific immune maturity evaluation based on continuous interval number medium operator. *Symmetry*.

[28] Liu Q., Hu H.-Y., Guo Y., Yang F.-X. (2019). Evaluation and decision making of organization quality-specific immunity based on MGDM-IPLAO method. *Open Physics*.

[29] Liu Q., Lian Z., Guo Y. (2020). Empirical analysis of organizational quality defect management enabling factors identification based on SMT, interval-valued hesitant fuzzy set ELECTRE and QRA methods. *Journal of Intelligent and Fuzzy Systems*.

[30] Liu Q., Lian Z., Guo Y., Tang S., Yang F. (2020). Heuristic decision of planned shop visit products based on similar reasoning method: from the perspective of organizational quality-specific immune. *Open Physics*.

[31] Liu Q., Lian Z., Guo Y., Yang F. (2020). Intuitively fuzzy multi-attribute group decision making of organizational quality specificity immune evolution ability based on evidential reasoning. *Journal of Intelligent and Fuzzy Systems*.

[32] Liu Q., Liang Y., Zhao D. Y., Guo Y. (2020). Influencing factors of organization quality-specific immune of intelligent manufacturing enterprises based on system dynamics simulation. *Dynamic Systems and Applications*.

[33] Liu Q., Kang X., Guo Y., Su Y., Shi L. P., Yang F. X. (2017). Influence mechanism of external social capital of university teachers on evolution of generative digital learning resources of educational technology of university teachers-Empirical analysis of differential evolution algorithm and structural equation model of Bootstrap self-extraction technique. *Eurasia Journal of Mathematics, Science and Technology Education*.

[34] Ma Q., Shi L., Hu L., Liu Q., Yang Z., Wang Q. (2016). Neural features of processing the enforcement phrases used during occupational health and safety inspections: an ERP study. *Frontiers in Neuroscience*.

[35] Yang Z. N., Wang Y. H. (2008). Construction of defense mechanism of organization health from the perspective of immune: a case study. *Nankai Business Review*.

[36] Nelson R. R., Winter S. G. (1985). *An Evolutionary Theory of Economic Change*.

[37] Birkinshaw J., Hood N. (2000). Characteristics of foreign subsidiaries in industry clusters. *Journal of International Business Studies*.

[38] Birkinshaw J., Ridderstråle J. (1999). Fighting the corporate immune system: a process study of subsidiary initiatives in multinational corporations. *International Business Review*.

[39] Jerne N. K., Frs M. D. (1985). The generative grammar of the immune system. *Bioscience Reports*.

[40] Jones A., Murphy J. T. (2011). Theorizing practice in economic geography: foundations, challenges, and possibilities. *Progress in Human Geography*.

[41] Liu Q. (2014). *Research on the Function Mechanism of Influencing Factors of Quality Defect Management on Quality Performance*.

[42] Lv P. (2011a). Research on the influence of geographical distribution of the relationships between knowledge sources and innovation on innovation performance. *Journal of Finance and Economics*.

[43] Lv P. (2011b). Empirical study on the influence mechanism of organizational immune behavior on organizational performance. *Science of Science and Management of Science and Technology*.

[44] Wang Y. H. (2007). Construction and operation mechanism of organizational immune system-A case study of Daya bay nuclear power station. *Science of Science and Management of Science and Technology*.

[45] Lv P., Wang Y. H. (2008). Research on enterprise adaptability from the perspective of organization immune. *Science Research Management*.

[46] Schmid S., Dzedek L. R., Lehrer M. (2014). From rocking the boat to wagging the dog: a literature review of subsidiary initiative research and integrative framework. *Journal of International Management*.

[47] Schweizer R., Lagerström K. (2019). “Wag the Dog” initiatives and the corporate immune system. *Multinational Business Review*.

[48] Shi L. P., Liu Q., Jia Y. Q., Yu X. Q. (2015). Optimization of quality performance improvement path based on projection pursuit-Raga-NK-GERT-An interpretation framework dominated by organization quality-specific immune and product life cycle. *Operations Research and Management*.

[49] Shi L. P., Liu Q., Jia Y. Q., Yu X. Q. (2014). Research on the relationships among network relationship intensity, total quality management practice and organizational learning-Expanding the potential path of organizational learning. *Management Review*.

[50] Shi L. P., Liu Q., Tang S. L. (2012). Study on quality performance improvement paths from the perspective of organization specific immune-An empirical analysis of projection pursuit method and enter method. *Nankai Business Review*.

[51] Shi L. P., Liu Q., Teng Y. (2015). Quality performance upgrading paths based on OSI-PP-Enter: theoretical framework and empirical analysis. *Journal of Industrial Engineering/Engineering Management*.

[52] Shi L. P., Liu Q., Wu K. J., Du Z. W. (2013). Function mechanism of organization quality-specific immune construction factor consistency on quality performance-An empirical analysis based on PP method, fit method and hierarchical regression analysis. *Industrial Engineering & Management*.

[53] Strutzenberger A., Ambos T. C. (2014). Unravelling the subsidiary initiative process: a multilevel approach. *International Journal of Management Reviews*.

[54] Winter S. G., Szulanski G. (2001). Replication as strategy. *Organization Science*.

[55] Yu J., Zaheer S. (2010). Building a process model of local adaptation of practices: a study of Six Sigma implementation in Korean and US firms. *Journal of International Business Studies*.

[56] Lv P., Wang Y. H. (2009). Study on organization immune behavior and mechanism. *Journal of Management*.

[57] Jiang T., Xiong W. (2017). Multi-layer distributed organization immune response model based on comprehensive perspective. *Science and Technology Management Research*.

[58] Xiong W., Feng X. B. (2012). Empirical study on the relationships between quality management practice and performance based on enterprise characteristic variables. *Journal of Zhejiang University*.

[59] Jiang T. (2015). *Research on the Effect Mechanism of Quality Management Practice on the Renewal of Organizational Operation Practice*.

[60] Yang Z. N., Li D. H. (2014). The dilemma of “new organization” and “small organization”: based on the defense mechanism of organization health from the perspective of immune. *Economics and Management*.

[61] Dai C. L., Ding X. S. (2013). Construction of enterprise internal control evaluation system based on organization immune theory. *Finance and Accounting Monthly*.

[62] Røvik K. A. (2011). From fashion to virus: an alternative theory of organizations’ handling of management ideas. *Organization Studies*.

[63] Wang Y. H., Lv P., Xu B. (2006). Study on organization immune. *Science of Science and Management of Science and Technology*.

[64] Nair A. (2006). Meta-analysis of the relationship between quality management practices and firm performance-Implications for quality management theory development. *Journal of Operations Management*.

[65] Chen L. J. (2014). *Research on the Evolution of R&D Industry Based on Self-Organization Theory*.

[66] Daft R. L., Weick K. E. (1984). Toward a model of organizations as interpretation systems. *Academy of Management Review*.

[67] Lv P. (2012). Enterprise ownership, internal and external knowledge network choice and innovation performance-An empirical study based on ICT Industry in China. *Studies in Science of Science*.

[68] Li Q. X., Sun P. S., Jin F. H. (2010). Research on supply chain quality management model based on immune perspective. *Commercial Research*.

[69] Kiesler S., Sproull L. (1982). Managerial response to changing environments: perspectives on problem sensing from social cognition. *Administrative Science Quarterly*.

[70] Porter M. E. (1985). *Competitive Advantage*.

[71] Ferrier W. J., Smith K. G., Grimm C. M. (1999). The role of competitive action in market share erosion and industry dethronement: a study of industry leaders and challengers. *Academy of Management Journal*.

[72] March J. G., Simon H. A. (1958). *Organizations*.

[73] Zhao Y. T. (2019). A probe into the development of urban morphology in Shapouwei Area of Fujian Province from the perspective of self-organization theory. *Architecture and Culture*.

[74] Ha K. (1989). *Higher Synergetics*.

[75] Qian X. S., Yu J. Y., Dai R. (1990). A new field of science-open complex giant system and its methodology. *Journal of Nature*.

[76] Wu J. C., Xie Y. P. (2017). Evolution and development of business ecosystem and dynamic analysis from the perspective of self-organization theory. *Enterprise Economy*.

[77] Ding Y., Li Z., Ge X., Hu Y. (2020). Empirical analysis of the synergy of the three sectors’ development and labor employment. *Technological Forecasting and Social Change*.

[78] Li T., Yang W., Li M. (2020). Engrailed 2 (EN2) acts as a glioma suppressor by inhibiting tumor proliferation/invasion and enhancing sensitivity to temozolomide. *Cancer Cell International*.

[79] Li B. Z., Zeng J. W., Wang D., Su Y. (2020). Research on co-evolution of enterprise green innovation system based on knowledge behavior. *Journal of Industrial Engineering/Engineering Management*.

[80] Liu X. Y., Wang J., Shan X. H. (2020). Research on the evolution dynamics of technological innovation network based on TERGMs. *Science Research Management*.

[81] Liu P., Mu D., Su J. (2015). Dynamics of resources integration in regional inland transportation system. *Journal of Systems Management*.

[82] Song Y. Q., Li H. J., Wang Q., Li G. J. (2020). Measurement and empirical research of synergy in complex systems based on Kolmogorov entropy. *Operations Research and Management Science*.

[83] Wang Z. Z., Tang Z. Y. (2021). Study on dissipative structure of regional innovation ecosystem. *Studies in Science of Science*.

[84] Zhang J. H., Chen Z. F., Ren Z. G., Yang L. X. (2020). Review on complexity science and application to economics: based on supported projects and related research. *Journal of Management Sciences in China*.

[85] Zhang L., Wang X. X., Li J. X. (2020). Dynamic evolutionary game of credit mechanism among core populations in E-commerce ecosystem. *Operations Research and Management Science*.

[86] Ali M. N., Husnine S. M. T. A. (2018). Solitary wave solution and conservation laws of higher dimensional zakharov-kuznetsov equation with nonlinear self-adjointness. *Mathematical Methods in the Applied Sciences*.

[87] Baig A. Q., Naeem M., Gao W. (2018). Revan and hyper-revan indices of octahedral and icosahedral networks. *Applied Mathematics and Nonlinear Sciences*.

[88] Dewasurendra M., Vajravelu K. (2018). On the method of inverse mapping for solutions of coupled systems of nonlinear differential equations arising in nanofluid flow, heat and mass transfer. *Applied Mathematics and Nonlinear Sciences*.

[89] Harraga H., Yebdri M. (2018). Attractors for a nonautonomous reaction-diffusion equation with delay. *Applied Mathematics and Nonlinear Sciences*.

[90] Owolabi K. M., Atangana A. (2019). Mathematical analysis and computational experiments for an epidemic system with nonlocal and nonsingular derivative. *Chaos, Solitons & Fractals*.

[91] Lv Z., Guo J., Lv H. (2022). Safety poka yoke in zero-defect manufacturing based on digital twins. *IEEE Transactions on Industrial Informatics*.

[92] Zhuang M., Zhu W., Huang L., Pan W.-T. (2021). *Research of Influence Mechanism of Corporate Social Responsibility for Smart Cities on Consumers’ Purchasing Intention, *.

[93] Li C., Wangchenxuan (2017). Green development assessment of smart city based on pp-bp intelligent integrated and future prospect of big data. *Acta Electronica Malaysia*.

[94] Tajuddin N. I., Abdullah R., Jabar M., Jusoh Y., Arbaiy N. (2017). Rasch model application in validating instrument for knowledge integration in small medium enterprises. *Acta Informatica Malaysia*.

[95] Zhang J. K., Luo W. D. (2010). Research on evolutionary dynamics of real estate industry based on self-organization theory. *East China Economic Management*.

[96] Zhang J. P., Shi X. M. (2019). Research on cooperative evolution mechanism of cloud logistics platform cooperation innovation system-Based on self-organization theory. *Journal of Jiaxing University*.

[97] Xu Q. J. (2003). A new probe into enterprise theory: enterprise self-organization theory. *Nankai Business Review*.

[98] Mi C., Shen Y., Mi W., Huang Y. (2015). Ship identification algorithm based on 3D point cloud for automated ship loaders. *Journal of Coastal Research*.

